The article "Exposure to Messages on Risk Factors for Noncommunicable Diseases in a Rural Province of Vietnam" was published in 2019. Journal: Biomed Res Int.

# Exposure to Messages on Risk Factors for Noncommunicable Diseases in a Rural Province of Vietnam

**DOI:** 10.1155/2019/7962947

**Published:** 2019-04-30

**Authors:** Bich Diep Pham, Bao Giang Kim, Thi Thu Huyen Nguyen, Van Minh Hoang

**Affiliations:** ^1^Institute for Preventive Medicine and Public Health, Hanoi Medical University, Hanoi, Vietnam; ^2^Hanoi University of Public Health, Hanoi, Vietnam

## Abstract

**Background:**

Providing messages on risk factors for noncommunicable diseases (NCDs) plays an important role in preventing disease.

**Objectives:**

This study investigated how often adults living in a rural area in northern Vietnam heard about risks factor for NCD and where they obtained that information.

**Methods:**

A cross-sectional survey was conducted using a multistage stratified cluster sampling to recruit 2970 participants. Data analyses were adjusted for all variables in a two-level multilevel Poisson regression model.

**Results:**

Overall, 77% of respondents had heard about NCDs, while 38.3 to 50% had been exposed to messages on risk factors of NCDs in the last month. Television, radio, and friends/neighbors were the most common sources of information. Most people exposed information no more than one or two sources. Factors associated with exposure to messages about risk were occupation, age group, education, and economic status.

**Conclusion:**

Intervention programs should focus on providing information primarily through television, considering influencing factors as well ensuring that messages reach target audiences.

## 1. Introduction

In recent years, noncommunicable diseases (NCDs), including cardiovascular diseases, diabetes, cancer, and chronic respiratory diseases, have appeared as key public health challenges, due to the high number of deaths they cause (38 million in 2012 or 68% of total deaths worldwide) [1, 2], expected to reach 52 million by 2030 [3]. NCDs are especially difficult problems for low- and middle-income countries (LMICs), considering the very high prevalence of NCDs in these regions [4]. In 2012, nearly three-quarters of NCD deaths occurred in LMICs [5], expected to increase by 20% by 2020 [4]. Among the causes of the increasing burden of NCDs in LMICs are industrialization, urbanization, economic development, and market globalization, all of which contribute to rapid changes in people's diets and lifestyles [6, 7]. Changes include a transition from traditional foods to high-fat/salt/sugar processed foods and from manual labour to physical inactivity [8]. Vietnam has recently been transformed from one of the world's poorest countries to a lower-middle-income country, typical of countries facing the challenge of NCDs. Since the economic and political reforms under Đ*ổ*i Mới in 1986, Vietnam has undergone rapid economic growth and development. The gross domestic product (GDP) per capita was 98 US$ per year in 1986 and had risen to 1333 US$ in 2010 (World Bank, 2015), among the fastest growth rates in the world [9]. There is a clear link between Vietnam's economic development and the increasing national burden of NCDs. The number of deaths due to NCDs in Vietnam rose from 288.000 in 2000 to 379.000 in 2010 [10]. In 2014, they were estimated to account for 73% of all deaths in Vietnam [1]. Together with economic development, behavioral risk factors for NCDs also increased, such as the harmful use of alcohol, unhealthy diets, and physical inactivity [11, 12]. For example, alcohol consumption by persons aged 15 years and older increased by 412%, from 1.6 liters in 1990 to 6.6 liters in 2010 [13, 14]. Additionally, a 2015 national survey revealed high prevalence for NCD risk factors, such as a lack of vegetable/fruit consumption among adults (57.2%), salt consumption (nearly twice what WHO recommends), and physical inactivity (28.1%) [15]. Since, according to WHO, a large proportion of NCDs can be prevented by reducing behavioral risk factors [1, 2], it is useful to explore the communication in the community about NCDs and NCDs' behavioral risk factors. Exposure to information about keeping healthy is reported to be associated with social determinants of health such as education level, employment status, or economic status, which may in turn affect choices about behavior related to NCDs [16–18].

The article "Exposure to Messages on Risk Factors for Noncommunicable Diseases in a Rural Province of Vietnam" was published in 2019. Journal: Biomed Res Int.

An understanding of the relationship between health communication outcomes and socioeconomic variables may help to develop a more effective prevention program. This paper describes the results of a study on exposure to health messages on NCDs for people in a rural province in Vietnam. The study also examined the relationship between socioeconomic variables and exposure to that health information.

## 2. Methods

### 2.1. Setting

This cross-sectional study was conducted in 2016 in Quoc Oai, a rural province located 20 km West of Hanoi, the capital of Vietnam. Quoc Oai district has one town and 20 communes that include both lowland and mountainous settings.

### 2.2. Sample Size and Sampling

The data used for this paper was obtained from a health system survey conducted in Quoc Oai in 2016 [19]. The sample size of that survey was estimated based on the WHO formula for estimating one population proportion in which* p* value is the expected proportion of households in the district incurring catastrophic expenditure, with an absolute precision of 1% and level of significance of 5%, resulting in a sample size of 1118 households. Since the study planned to use the cluster sampling technique, the design effects of 2 and nonresponse rate of about 10% were applied, giving a final sample size of 2400 households. A multistage stratified cluster sampling approach was applied to select the 2400 households. Firstly, two strata (lowland and mountain) were selected. In each stratum, 21 clusters in the lowland area and 9 clusters in the mountainous area were selected. In each cluster, 80 households were selected using a simple random sampling technique.

The article "Exposure to Messages on Risk Factors for Noncommunicable Diseases in a Rural Province of Vietnam" was published in 2019. Journal: Biomed Res Int.

The interviews on household characteristics were done with the heads of the selected households. The interviews on self-reported health problems, including chronic noncommunicable diseases, were done with up to two people per household (one person aged 15 -59 years old and one person aged 60 years old and above). The sections of people for interviews on self-reported health problems were done using Kish method [20].

### 2.3. Questionnaire

The results reported here are taken from a larger questionnaire used in a health system survey (this part only shows those questions used in this study). The first part comprised questions about social economic variables: sex, age, education, occupation, ethnicity, religion, household permanent and durable properties, and location. The household location (plains or mountain) was identified based on the sampling sheet and location of the house. Some variables were recoded into fewer categories for the analysis as our interest. Age group was recoded into two categories: from 15 to 59 years and 60 and above because the younger and older groups might be exposed to different information sources. Occupation was recoded into three categories: retired group who have health insurance; farmer group, accounting for nearly half the sample and who mostly do not have health insurance; and other occupations. Household wealth index was calculated based on the household permanent and durable properties. The index was divided into quintiles, with the first quintile as the poorest and the fifth as the richest.

The second part of the questionnaire concerned the question: “Have you ever heard about noncommunicable diseases such as hypertension, diabetes, cancer, COPD, asthma?” Those who answered “yes” continued to answer the following questions. Four detailed questions were: “Have you ever heard that smoking, abusing alcohol, high-fat/sugar/salt diet and physical inactivity increase the risk of getting NCDs.” The answers were “no” and “yes” and all people who answered “yes” were asked to provide the number of times they had heard about the risk of getting NCDs by each of four risk factors (smoking, abusing alcohol, high-fat/sugar/salt diet, and physical inactivity). Questions were also posed about the sources of information, which might include television, radio, friends/neighbors, family members, health workers, internet, newspapers/magazines, books, leaflets, posters, and others.

The article "Exposure to Messages on Risk Factors for Noncommunicable Diseases in a Rural Province of Vietnam" was published in 2019. Journal: Biomed Res Int.

### 2.4. Data Collection

The questionnaire was piloted in Quoc Oai province to make sure the meaning and words of the questions were understandable and then revised to increase clarity. Twelve investigators were trained during one week to collect the data, to ensure that they understood all the questions and would give the same explanation to interviewees.

Data was collected during face-to-face interviews. Each investigator had names on the list of respondents and made appointments with them in their homes. Once there, the investigators explained the purpose of the study and invited the respondents to participate. Oral consent was given before the interviews began. The investigators asked each question and filled in the answers provided on the data sheets. Supervisors reviewed the data collected. All of the 2970 people invited to participate did agree to be interviewed.

### 2.5. Data Analysis

The analysis was performed with SPSS for Windows (version 20) and STATA (version 15). Descriptive statistics were used to determine the frequency and percentage of having heard messages on NCDs and on risk factors for NCDs. The numbers exposed to messages on risk factors for NCDs were calculated and used as the dependent variable in the two-level multilevel Poisson regression model. The dependent variable was a count variable with a value from 0 to 4 (0: did not hear of any risk factor that causes NCDs in the past month; 1: heard of one factor; and 4: heard of 4 factors).

A two-level multilevel Poisson regression model was used to investigate the relationship between the numbers exposed to messages on risk factors of NCDs and independent variables. Individuals (level 1) were nested within cluster (level 2). Two models were fitted. Model 1 included the individual level variables (occupation, education, age group, and household wealth index). Model 2 included individual level and cluster level variables that took into account clustering of the data. The results are presented as the prevalence ratio (PR) with 95% confidence intervals (95% CI).

### 2.6. Ethics

This study was approved by the Scientific and Ethical Committee for Biomedical Research, Hanoi School of Public Health. All respondents were invited to participate in the interview and informed about the objectives and purpose of the study; it was made clear to participants that they had the right to continue or withdraw from the study whenever they wished.

The article "Exposure to Messages on Risk Factors for Noncommunicable Diseases in a Rural Province of Vietnam" was published in 2019. Journal: Biomed Res Int.

## 3. Results 

Table 1 shows the general characteristics of the study sample. There were more women and men in the study. Nearly half of respondents were farmers. The proportions of respondents who were of high school or lower level of education and aged from 15 to 59 years old accounted for 87% and 73% of total (respectively).

### 3.1. People Who Had Heard about NCDs

Among the 2970 people interviewed, 2281 (77%) had heard about NCDs such as hypertension, diabetes, cancer, COPD, and asthma; 183 (6.2%) had not heard about any of the four main lifestyle risk factors for NCDs, and 942 (31.7%) had heard about all four main factors (data not shown).

The data in Table 2 shows that most people (55.0% to 65.7%) who had heard about NCDs knew the four main lifestyle risk factors for NCDs (smoking, alcohol abuse, diet high in fat/salt/sugar, and physical inactivity). Less than half of them had heard such information during the past month before the interview.

### 3.2. Sources of Information on Risk Factors for NCDs

In general, the greatest proportion of respondents reported having been exposed to information about risk factors for NCDs through television (Table 3, 67.4% - 78.1%), followed by radio with messages related to smoking; by friends/neighbors with messages related to drinking, diet, and inactivity. Family members, health workers, internet, and others including newspapers, leaflets, and posters were reported by much lower proportions of respondents.

However, a greater proportion of older people (60 years and above) was exposed to information about risk factors for NCDs, especially related to diet and inactivity, from friends/neighbours and health workers, whereas for those among younger people (from 15 to 59 age) the greatest exposure was from Internet websites.

More than half of the people said that they were exposed to information from one source but about one-third got information from two to three sources and very few (less than 1%) made use five different sources (Table 4).

People reported exposure to messages on each risk factor for NCDs during the past month from 2.7 to 3.3 times; notably, they had heard smoking-related messages 3.3 times and were exposed to messages related to physical inactivity 2.7 times.

### 3.3. Factors Associated with Exposure to Number of Messages on Risk Factors for NCDs

Table 5 reports the results from a set of multilevel Poisson regression models using prevalence ratios (PR) and 95% CI.

The model 1 of one level (individual level) and model 2 of two levels (both individual and cluster level) remained significant in models, suggesting that individual and cluster level factors were important for predicting the numbers of messages on risk factors in the past month. Model 1 shows that four factors: occupation, age group, education, and household wealth index were significantly associated with the number of messages on risk factors to which they were exposed. Being farmers and being retired, increased the frequency by 1.15 and 1.38 times (respectively) of having heard one message, compared to other occupations. People aged from 15 to 59 years had an increased frequency, by 1.09 times, of having heard one message, compared to people of 60 years or more. Those whose education was to university and higher levels had increased frequency, by 1.38 times, of having heard one message, compared to those with high school or lower level. With regard to household wealth index, the rich and richest groups were more likely to have heard messages on risk factors for NCDs from 1.21 and 1.33 times compared to the poorest.

The article "Exposure to Messages on Risk Factors for Noncommunicable Diseases in a Rural Province of Vietnam" was published in 2019. Journal: Biomed Res Int.

However, in Model 2 with both individual and cluster levels, being a farmer not significantly associated with the numbers of messages on risk factors, while belonging to the group of the third quintile (the average group) was significantly associated.

## 4. Discussion

The first issue identified by this study is that there is still a large proportion, nearly one-quarter, of the population who have never heard about NCDs. More than half of those who had heard about NCDs were aware of four lifestyle risk factors, principally smoking and alcohol abuse, but also diet and lack of physical activity. The main source of information about NCD risk factors was the television, much higher than alternatives such as radio and friends/neighbors. Having exposure to health messages on the four lifestyle risk factors was also related to demographic variables such as occupation, education, and economic status. The finding that many people were exposed to messages about the main lifestyle risk factors may be a result of the Vietnam NCD prevention and control programme [21]. Among the four lifestyle risk factors, the most well-known among the respondents were drinking and smoking. The two most often mentioned sources of information for messages on smoking were television and radio, while for messages on the three other lifestyle risk factors, television and friends/neighbors were more often noted. This result may reflect the activity of the Vietnam Steering Committee on Smoking during recent years to provide messages about tobacco through many channels, especially mass media channels like television and radio.

The observation that television was the main source of information on risk factors confirms the important role for mass media, especially television. Following television, the older people were most exposed to messages through friends/neighbors and health workers, whereas younger people's exposure was more through friends/neighbors and Internet. This finding is similar to that from a study in Japan, where people were exposed to health information mostly through television (51.1%), followed by friends and relatives (34.0%) and newspapers (31.4%) [22]. However, in Hong Kong, the most popular channel through which people sought health information at least one a month was from newspapers/magazines (66.2%), television (61.4%), radio (35.6%), or Internet (33.2%) [23]. In both of these studies, Internet was the most popular channel among younger people than older people, similar to the results in our study. A study in Nigeria had different results; there, health workers were the most popular channel for sourcing medical information (64.4%), followed by books (36.2%) and mass media (28.8%) [24]. The difference in preference of sources from country to country might depend on the trust of people in the different channels, the quality of information from each channel, and the availability of the equipment. In Vietnam, a review of the information and communications technology sector and E-health estimated that in 2010, 18 million households, or 90% of the population, had exposure to television sets [25]. Besides television, radio is highly accessed, especially the Voice of Vietnam, the official network of the Vietnamese Government, with 61 provincial radio stations, and broadcasts on AM, FM, and shortwave throughout the country. This coverage may explain why both television and radio were key sources of information. On the other hand, in Vietnam, 99% of communities have a health station and 79% of villages have active village health workers [26], but the role of health workers in communicating with the public about NCDs and risk factors seems more frequent among older people but not younger ones. This might be due to deficiencies in human resource numbers in rural Vietnam [27]. Another result from this sample was published separately, showing that older people with noncommunicable diseases utilized health care services more than younger ones [19]. Therefore, this might suggest the evidence that the health workers passively provided information about risk factors of NCD for older people through face-to-face counseling, when they met people in their health working places.

The article "Exposure to Messages on Risk Factors for Noncommunicable Diseases in a Rural Province of Vietnam" was published in 2019. Journal: Biomed Res Int.

Four socioeconomic factors were found to be associated with exposure to messages on NCD risk factors: occupation, education, age group, and economic status. Similar results have been reported from both developed countries such as Japan [22], Hong Kong [23], and the US [28] and in other developing countries as Nigeria [24]. Apparently, the higher the level of education, the younger the age and higher the economic status, the better the exposure to health information. The results were consistent with findings from studies in Japan and Hong Kong [22, 23]. A study in the US also showed that the highest income group was more likely to seek cancer information [28]. However, studies in China did not find a relationship between health knowledge levels and income [29]. We also found that retired people were more likely to have been exposed to messages on NCD risk factors compared to other occupations. It is possible that this finding is related to the popularity of television and radio as sources of information and to the fact that retired people had more free or flexible time to use these sources. Additionally, retired people belong to the elderly group which may be likely to increase their attention to a healthy lifestyle to promote and prolong life. Retired people also had health insurance, which makes it easier for them to utilize health care services [19]. The results of this study also support the above explanation that after television, the second channel that exposed older people to messages on diet and inactivity were health workers.

In summary, our findings reveal that the messages related to NCD risk factors were exposed to more than half of community people through different channels. The important social determinants, particularly occupation, education, age group, and economic status, that have been found to influence health outcomes are also strongly linked to exposure to NCD health communication messages. The data also suggested evidence for inequality in health communication in the rural North of Vietnam, which also has been found in other countries.

Providing greater access by taking into account factors associated with social determinants may contribute to addressing social disparities in health communication. For example, television should continue to be used to deliver messages on NCD prevention and control, to reach a large proportion of the population. Health commune centers should provide training for village health workers so that they can actively and directly access the disadvantaged groups such as the poor and poorest groups or those with lower education levels to communicate important health messages related to NCDs.

## 5. Study Limitations

The participants in this study came from one province in Vietnam, which although it is a typical area for the rural North does not make it representative for the whole country. As the data were collected in a cross-sectional study, they can only reveal associations between health communications outcomes and socioeconomic variables, but no potential causal links.

The article "Exposure to Messages on Risk Factors for Noncommunicable Diseases in a Rural Province of Vietnam" was published in 2019. Journal: Biomed Res Int.

## 6. Conclusions 

NCDs are estimated to account for 73% of all deaths in Vietnam, which makes exposure to messages on risk factors of NCDs an important item for prevention and control programs. Our findings suggest that programs emphasize television and radio messages which are popular and can reach a large population. Special efforts are needed to reach disadvantaged groups such as older people, the less educated, and those with lower economic status, which we found to have less exposure to messages.

## Figures and Tables

**Table 1:** General characteristics of the study sample (n= 2970).

Variables	n	%
Gender		

Male	1331	48.8

Female	1639	55.2

Occupation		

Retired	137	4.6

Farmer	1420	47.8

Others^a^	1413	47.6

Location		

Plains (21 lowland clusters)	2120	71.4

Mountainous (9 mountainous clusters)	850	28.6

Education		

High school or lower	2585	87.0

University/higher	385	13.0

Household wealth index		

1st quintile-Poorest	597	20.1

2nd quintile-Poor	571	19.2

3rd quintile-Average	601	20.2

4th quintile-Rich	595	20.0

5th quintile- Richest	606	20.4

Age		

15-59 years	2168	73.0

60 years and above	802	27.0

Age (Mean; SD)	46.3; 18.7	

^a^included government staff, small traders, army, providing personal services, providing social services, etc.

**Table 2:** NCD-related Information that 2970 people had been exposed to.

Information	Had ever heard		Heard within past month	
	n	%	n	%
Smoking increases the risk of getting NCDs.	1945	65.5	1455	49.0

Abusing alcohol increases the risk of getting NCDs.	1950	65.7	1486	50.0

High fat/salt/sugar diet increases the risk of getting NCDs.	1819	61.2	1277	43.0

Physical inactivity increases the risk of getting NCDs.	1634	55.0	1138	38.3

**Table 3:** Information sources for those exposed to NCD information in past month, by four lifestyle risk factors for NCDs, and by age group.

Information sources	Smoking						Drinking						Diet						Inactivity					
	< 60 age (n = 1096)		>= 60 age (n= 359)		Total (n = 1455)		< 60 age (n = 1112)		>= 60 age (n= 374)		Total (n = 1486)		< 60 age (n = 940)		>= 60 age (n= 337)		Total (n = 1277)		< 60 age (n = 814)		>= 60 age (n= 324)		Total (n = 1138)	
	n	%	n	%	n	%	n	%	n	%	n	%	n	%	n	%	n	%	n	%	n	%	n	%
Health workers	119	10.9	62	17.3	181	12.4	115	10.3	61	16.3	176	11.8	133	14.1	93	27.6	226	17.7	80	9.8	68	21.0	148	13.0

Family members	118	10.8	39	10.9	157	10.8	148	13.3	56	15.9	204	13.7	74	7.9	36	10.7	110	8.6	69	8.5	43	13.3	112	9.8

Friends/neighbor	218	19.9	66	18.4	284	19.5	259	23.3	88	23.5	347	23.4	161	17.1	71	21.1	232	18.2	140	17.2	85	26.2	225	19.8

Radio	222	20.3	81	22.6	303	20.8	227	20.4	86	23.0	313	21.1	136	14.5	52	15.4	188	14.7	126	15.5	50	15.4	176	15.5

TV	855	78.0	282	78.6	1137	78.1	841	75.6	289	77.3	1130	76.0	664	70.6	236	70.0	900	70.5	556	68.3	211	65.1	767	67.4

Internet	184	16.8	4	1.1	188	12.9	173	15.6	4	1.1	177	11.9	164	17.4	5	1.5	169	13.2	152	18.7	3	0.9	155	13.6

Others^*∗*^	134	12.2	30	8.3	164	10.6	93	8.4	26	6.9	119	8.0	100	10.6	23	6.8	123	9.6	85	10.4	26	8.0	111	9.7

^*∗*^newspaper, leaflet, poster, etc.

The article "Exposure to Messages on Risk Factors for Noncommunicable Diseases in a Rural Province of Vietnam" was published in 2019. Journal: Biomed Res Int.

**Table 4:** Number of information sources and times that people were exposed to NCD information in past month by four lifestyle risk factors.

Number of information source and times	Smoking (n = 1455)		Drinking (n = 1486)		Diet (n = 1277)		Inactivity (n=1138)	
	n	%	n	%	n	%	n	%
One source	808	55.5	798	53.7	794	62.2	718	63.1

Two sources	424	29.1	471	31.7	341	26.7	309	27.2

Three sources	153	10.5	157	10.6	105	8.2	82	7.2

Four sources	53	3.6	42	2.8	27	2.1	21	1.8

At least five sources	19	0.9	17	1.0	9	0.8	5	0.5

	Mean	SD	mean	SD	mean	SD	mean	SD

Number of times exposed to information in last month	3.3	4.5	3.0	4.0	2.7	3.8	2.7	4.0

SD: Standard deviation

**Table 5:** NCD risk factor message exposure in relation to socio-demographic variables.

Variables	Model 1		Model 2	
	PR	95%CI	PR	95%CI
*Fixed effects*				

*Individual characteristics*				

Occupation (other^a^: ref)	1		1	

Retired (0)	1.58	1.41 – 1.79^*∗∗∗*^	1.38	1.22 – 1.56^*∗∗∗*^

Farmer (1)	1.15	1.08 – 1.22^*∗∗∗*^	1.05	0.99 – 1.213

Age groups (60 and above: ref)	1		1	

From 15 to 59 years	1.09	1.02-1.16 ^*∗∗*^	1.12	1.04-1.19^*∗∗*^

Education (high school or lower: ref)	1		**1**	

University/higher	1.38	1.28-1.50^*∗∗∗*^	1.24	1.15-1.35^*∗∗∗*^

Household wealth index (1st quintile-Poorest: ref)	1		1	

2nd quintile -Poor	1.04	0.95-1.14	1.07	0.98-1.12

3rd quintile -Average	1.04	0.96-1.14	1.13	1.03-1.24^*∗*^

4th quintile-Rich	1.21	1.11-1.32^*∗∗∗*^	1.23	1.12-1.36^*∗∗∗*^

5th quintile- Richest	1.33	1.22-1.46^*∗∗∗*^	1.40	1.27-1.54^*∗∗∗*^

*Random effects*				

*Cluster variable*				

Estimate			0.2 (0.12-0.35)	

Variance (SE)			0.06	

Log likelihood	-5476.61		-5132.27	

LR test vs. Poisson (p)	0.000		0.000	

^a^ included government staff, small traders, army, providing personal services, providing social services, etc. PR: Prevalence Ratios after adjusting for other factors in the model;

CI: Confidence interval;  ^*∗*^*p* < 0.05;  ^*∗∗*^*p* < 0.01  ^*∗∗∗*^*p* < 0.001;

## Data Availability

The data used to support the findings of this study may be released upon application to the [Scientific Committee Board at Hanoi University of Public Health] for consideration, who can be contacted at [phambichdiep@hmu.edu.vn and hvm@huph.edu.vn].

The article "Exposure to Messages on Risk Factors for Noncommunicable Diseases in a Rural Province of Vietnam" was published in 2019. Journal: Biomed Res Int.

## Abbreviations

NCDs: Noncommunicable diseases
LMICs: Low- and middle-income countries
GDP: Gross domestic product
WHO: World Health Organization
COPD: Chronic obstructive pulmonary disease.

## Additional Points

*Key Messages.* (i) Most people knew about NCDs and had been exposed to information on lifestyle risk factors for NCDs, mainly from television, radio, and friends/neighbors. (ii) Socioeconomic factors influenced exposure to the messages. (a) Retired people were more likely to be exposed to messages than were other occupations. (b) Younger people were more likely to be exposed than older ones. (c) High school and lower education level were less likely to be exposed than above high school education level. (d) People with higher economics status were more likely to be exposed to the messages than the poorest.
